RETRACTED

# The Inhibitory Effect of Doxycycline on Cisplatin-Sensitive and -Resistant Epithelial Ovarian Cancer

**DOI:** 10.1371/journal.pone.0089841

**Published:** 2014-03-05

**Authors:** Wei Wu, Li-hua Yu, Bei Ma, Ming-juan Xu

**Affiliations:** 1 Department of Gynecology and Obstetrics, Changhai Hospital, Second Military Medical University, Shanghai, P.R.China; 2 Department of Physiology, Second Military Medical University, Shanghai, P.R.China; Yong Loo Lin School of Medicine, National University of Singapore, Singapore

## Abstract

**Background:**

Detecting a new effective and hypotoxic anticancer drug is an emerging new strategy for cancer chemotherapy. Doxycycline (DC) is a kind of antibiotics but also inhibits tumorigenesis.

**Methods:**

MTT and cell invasion assay, flow cytometry, western-blot analysis and nude mice were used to investigate the effects and underlying mechanisms of doxycycline on epithelial ovarian cancer cells.

**Results:**

Doxycycline inhibited the proliferation and invasion of SKOV3 and SKOV3/DDP; induced moderate apoptosis of SKOV3/DDP. CXCR4 expression at both mRNA and protein levels was downregulated in both cell lines when treated with doxycycline. Akt and ERK1/2 were involved in doxycycline effect on cell proliferation of SKOV3 but not of SKOV3/DDP. Akt and EKR1/2 phosphorylation were activated by SDF-1α, which was then inhibited by doxycycline in SKOV3. Pro-caspase-3 expression was significantly higher in SKOV3 than that in SKOV3/DDP which was upregulated when treated with doxycycline. In vivo, doxycycline inhibited peritoneal tumor xenograft and decreased malignant ascites.

**Conclusion:**

Doxycycline not only has an inhibitory effect on ovarian cancer, but also can increase sensitivity to cisplatin. SDF-1α/CXCR4-regulated Akt and ERK 1/2 activations are probably involved in the antitumor effect of doxycycline on SKOV3 cells, while upregulation of pro-caspase-3 may be the main mechanism involved in SKOV3/DDP cells.

## Introduction

Epithelial ovarian cancer (EOC) accounts for over 90% of all ovarian malignancies and is primarily a disease of postmenopausal women, occurring most commonly in sixth and seventh decades of life [1]. It represents the most common cause of death among women with gynecologic malignancies and the overall 5-year survival rate is only 30% [2].

At present, standard treatment for ovarian cancer involves tumor debulking and platinum-based chemotherapy [3]. The response to this regime is at least 70% of cases, however, 60–80% of first responders will relapse within 18 months with a platinum-resistant disease [4].

Cisplatin (DDP), a noncycle-dependent cytotoxic platinum derivative, has been frequently used in different solid tumors, including gastric, testicular, urologic, head, neck, and ovarian cancer [5]. Platinum compounds exert their cytotoxic effect by forming intrastrand platinum-DNA cross-links. This inhibits DNA replication and ultimately leads to apoptosis [6]. However, like other anticancer drugs, cisplatin-resistance remains a significant obstacle to its clinical success. Most patients with recurrent ovarian cancer will eventually develop platinum-resistant disease [7], making tumor cells refractory to therapy. Therefore, it is necessary to seek new economic and effective chemotherapy drugs which have antitumor activities and/or increase antitumor responses to platinum-based chemotherapy.

RETRACTED

Doxycycline (DC) is a kind of second-generation tetracyclines which is commonly used to treat a variety of infections. Current studies have demonstrated that doxycycline is a pluripotent drug that affects many anticarcinogenic functions, including anti-tumor growth effect on human oral squamous-cell carcinoma and inhibition of migration of melanoma cells [8]–[9]. Doxycycline also has a potential for enhanced therapeutic activity of biological cancer therapies [10]. However, the effect of doxycycline on epithelial ovarian cancer cells and the underlying mechanisms remain unknown.

Therefore, in our experiment, we aim to demonstrate that doxycycline has an anticancer activity on epithelial ovarian cancer cells, and to further explore the underlying mechanisms involved.

## Materials and Methods

### Ethics statement

This study was carried out in strict accordance with the recommendations in the Guide for the Care and Use of Laboratory Animals of the National Institutes of Health. All procedures in this study were approved by the Institutional Animal Care and Use Committee of Second Military Medical University. All surgery was performed under sodium pentobarbital anesthesia, and all efforts were made to minimize suffering.

### Cell culture and reagents

Human ovarian cancer cell lines HO8910 was obtained from department of pathophysiology of Second Military Medical University. SKOV3 and its cognate cisplatin-resistant cells SKOV3/DDP were obtained from ATCC (American Tissue Culture Collection). SKOV3.ip cells were provided by the Department of Gynecology and Obstetrics, Shanghai First People's Hospital (obtained from ATCC). Cells were maintained in RPMI-1640 medium with 10% fetal bovine serum at 37°C in a humidified 5% CO_2_ atmosphere. Cisplatin, doxycycline, SDF-1α, antibody against β-actin were purchased from Sigma-Aldrich. Antibodies against CXCR4, phosphor-Akt, total Akt, phosphor-ERK, total ERK, MMP-2, MMP-9, caspase-3 were purchased from Cell Signaling Technology. Transwell kit was purchased from BD, USA. ELISA kit was purchased from R&D, USA. Cell apoptotic kit was purchased from Roche, USA. Small interfering RNAs were synthesized by Genepharma Company (Shanghai, China). Xfect Transfection Agent was purchased from Clontech, USA. RNeasy minikit was purchased from QIAGEN, Clifton Hill, Australia.

RETRACTED

### MTT assay

As we reported before^11^, the MTT (methylthiazoltetrazolium) assays were conducted to assess cell viability. Cells suspension were seeded in 96-well plates after 12 h for attachment then treated with different concentrations of cisplatin or doxycycline. Drug-treated cells were incubated for 48 h and then 5 mg/ml MTT solution was added to the cultures for an additional 3–4 h. Finally, the medium containing MTT was aspirated off and 100 µl DMSO solution was added. As a result, living cells formed crystals due to the presence of MTT. Crystals were dissolved by DMSO and the absorbance was measured at 490 nm by an immunosorbent reader.

### Real-time PCR

Total RNA was isolated using a RNeasy minikit (QIAGEN, Clifton Hill, Australia). Two µg total RNA was reversely transcribed to cDNA in a 25-µl reaction containing 15 nmol/L MgCl2, 375 mmol/L KCl, 50 mmol/L dithiothreitol, 250 mmol/L Tris-HCl (pH 8.3), 10 mmol/L all four dNTPs, 20 U RNase inhibitor, 200 U M-MLV reverse transcriptase, and 50 ng oligo18 primer. The mixture was incubated at 70°C for 5 min and then at 42°C for 60 min followed by 10 min at 70°C. The following primers were used: CXCR4, 5-CCAACGTCAGTGAGGCAGAT-3 (forward) and 5-GGCAGGATAAGGCCAACCAT-3 (reverse); β-actin, 5-GTGGGGCGCCCCAGGCACCA-3 (forward) and 5-CTCCTTAATGTCACGCACGATTTC-3 (reverse). Real-time PCR was carried out using Rotor-Gene 3000 (Corbett Research, Sydney, Australia) in a 25-µL reaction mixture. 2× Taq PCR master mix and 0.2 µmol/L each primer were used. Real-time PCR conditions were optimized according to preliminary experiments to achieve a linear relationship between RNA concentration and PCR products. The specificity of the primers was verified by examining the melting curve as well as subsequent sequencing of the real-time RT-PCR products. Distilled water was used in place of cDNA as a negative control. All samples were normalized against internal β-actin control. Gene expression was calculated using the comparative threshold cycle (Ct) method.

### Western-blot analysis

As we reported previously [11], cells were harvested and homogenized in cold lysis buffer (50 mM Tris-HCl, pH 7.4, 150 mM NaCl, 1% Triton X-100, 1% deoxycholic acid sodium salt, 0.1% SDS, and a protease inhibitor mixture) using a homogenizer. Total protein concentration was determined by the Bradford method using bovine serum as a standard. Equal amounts of proteins were separated by 10% SDS-PAGE and transferred to polyvinylidene difluoride membranes. After blocked in blocking buffer consisting of 20 mM Tris-HCl, Ph 7.4,137 mM NaCl, 0.1% Tween 20, and 5% nonfat milk for 2 h at room temperature, membranes were incubated overnight at 4°C in primary antibody (anti-β-actin 1∶1000, anti-CXCR4 1∶1000, anti-phosphor-Akt 1∶1000, anti-total-Akt 1∶1000, anti-phosphor-ERK 1∶1000, anti-total-ERK 1∶1000, anti-MMP-2 1∶1000, anti-MMP-9 1∶1000). The blots were then incubated with HRP-conjugated secondary antibody (1∶1000, Santa Cruz) for 2 h at room temperature, and finally visualized in ELC solution. For 1 min and exposed onto Kodak film for 1–30 min. For control of correct gel loading, β-actin quantification was used. To quantify Western blot signals, band density was measured using UMAX PowerLook III and normalized with respect to the control.

RETRACTED

### ELISA assay

The amounts of SDF-1 in the conditioned media were determined using sandwich ELISA (sensitivity 15 pg/ml) according to manufacturer's protocols.

### Cell invasion assay

SKOV3 and SKOV3/DDP cell invasions were evaluated using 24-well transwell cell culture chambers with 8.0 µm pore polycarbonate filter inserts. The filters were firstly coated with BD matrigel. The stock solution of matrigel was diluted using serum-free RPMI-1640 medium (1∶1). An amount of diluted matrigel was painted into each filter insert and stayed at room temperature for 10–15 minutes to dry. Then, cultured cells were trypsinized and suspended in serum-free RPMI-1640 medium at a concentration of 2×10^5^ ml. A total of 500 µl of 10% FBS/RPMI-1640 medium or 500 µl of 50 ng/ml SDF-1 solution was added to the lower chamber and 100 µl cell suspension was applied to coated insert filters. The chamber was incubated for 3 h to allow cell attachment then cells were treated with doxycycline. The chamber was incubated for 36 h to allow cell invasion; the insert was then fixed with dehydrated alcohol for 15 minutes, and then stained with 0.1% crystal violet for 15 minutes and washed with 1×PBS. The unneeded cells on the upper or lower side of filter were scraped. The membrane was mounted on a slide and then examined under a microscope using 20× magnification. Invasion was quantified by measuring the stained cells in three random areas per membrane.

### Flow cytometric analysis of cell apoptosis

Cells were collected and double stained with phycoerythrin-conjugated Annexin V and PE according to the manufacturer's instructions. Annexin V–positive cells were considered apoptotic, and their percentage of the total number of cells was calculated. Ten thousand events were collected for each sample using a Becton Dickinson FACScan (Flow Cytometry Facility, Roswell Park Cancer Institute, Buffalo, NY), and data were analyzed using the Winlist program (VeritySoftware House, Topsham, ME).

RETRACTED

### siRNA transinfected technology

The target sequences for ERK were 5′- GUGCUCUGCUUAUGAUAAUTT-3′ (sense) and 5′- AUUAUCAUAAGCAGAGCACTT -3′ (antisense). AKT siRNA were: 5- GACGGGCACAUUAAGAUCATT-3 (sense) and 5- UGAUCUUAAUGUGCCCGUCTT -3 (antisense). Scramble siRNA duplexes were designed (5- UUCUCCGAACGUGUCACGUTT -3 and 5- ACGUGACACGUUCGGAGAATT -3) as a negative control (NC). Cells were transfected with 25 nM target siRNAs or control siRNA using Xfect Transfection Agent according to the manufacturer's instructions, and transfection was carried out for 24 hr (for AKT and ERK). Subsequently, the culture medium was replaced with 1640 medium supplemented with 10% heat-inactivated FBS. After 48 h, MTT assays were conducted to assess cell viability.

### Peritoneal tumor xenograft in nude mice

Nude (BALB/c-nu) mice (4 weeks, 18–20 g, provided by Chinese Academy of Science, BeiJing) were divided into three groups: a control group, a tumor group and a doxycycline-treated tumor group. For the tumor group, we injected SKOV3.ip cells to the mice peritoneal cavity at a density of about 8×10^6^/ml. The cells were resuspended in 400 µl serum-free RPMI-1640 medium and then injected. For the doxycycline-treated tumor group, after injected tumor cells for 14 days, doxycycline (3 mg/mouse) was i.p. injected everyday to suppress tumor growth. For the control group, mice were treated with equal volume of PBS. All mice were killed at day 21 after the first injection. Mice weight, tumor sizes and ascites were evaluated in all three groups.

### Statistical analysis

All data are shown as mean ± S.E.M. Experiments were independently done three times. Unpaired Students' test was used for two groups of data. One way ANOVA was used for multiple comparisons (SPSS software version 16.0), P-values<0.05 was considered as statistically significant.

## Results

### Doxycycline inhibits proliferation of epithelial ovarian cancer cells

After 48 h treatment with cisplatin and doxycycline in different concentrations, cell viability was decreased in a dose-dependent manner in HO8910 (Fig. S1A, B), SKOV3 (Fig. 1A, C) and SKOV3/DDP (Fig. 1B, D). The IC_50_ of doxycycline in SKOV3 was compared with that in SKOV3/DDP. The results showed that the IC_50_ was 16.33 µg/ml in SKOV3 (Fig. 1C) and 8.53 µg/ml in SKOV3/DDP (Fig. 1D) respectively, which indicated that SKOV3/DDP cells were more sensitive to doxycycline treatment than SKOV3 cells.

RETRACTED

**Figure 1:** MTT tests showing the viability of ovarian cancer cells incubated with indicated concentrations of cisplatin and doxycycline for 48 SKOV3 (A, C) and SKOV3/DDP (B, D) cell viability was inhibited in a dose-dependent manner by treatment with cisplatin and doxycycline. E, F showed that co-treatment with cisplatin (1.5 µg/ml and 2.5 µg/ml) and doxycycline (10 µg/ml) had a significant growth inhibition in SKOV3 cells compared with that of cisplatin or doxycycline treated alone. G, H showed that when combined doxycycline (2.5 and 5 µg/ml) with different concentrations of cisplatin, the IC_50_ of cisplatin in SKOV3/DDP cells was 3.36 and 2.66 µg/ml respectively. n = 9. *, *p*<0.05; **, *p*<0.01.

### Doxycycline sensitizes ovarian cancer cells to cisplatin

We conducted experiments with co-application of cisplatin and doxycycline. Firstly we selected two low doses (1.0 and 1.5 µg/ml) of cisplatin and combined them with low-dose doxycycline (0–10 µg/ml) respectively. In HO8910 cell line, a significant inhibition of cell growth was observed 48 hours after co-application of 1.0 µg/ml (Fig. S1C) or 1.5 µg/ml (Fig. S1D) cisplatin with 7.5 or 10 µg/ml doxycycline, while cisplatin treated alone lacked the effect. The similar results were shown in SKOV3 cell line, with a significant inhibition of cell growth when combining 1.5 µg/ml (Fig. 1E) or 2.5 µg/ml (Fig. 1F) cisplatin with 10 µg/ml doxycycline. Next, we selected two doses (2.5 and 5 µg/ml) of doxycycline and combined them with different concentrations of cisplatin (0–100 µg/ml), respectively. The IC_50_ of cisplatin in the presence of doxycycline (2.5 and 5 µg/ml) was 3.36 µg/ml and 2.66 µg/ml, respectively (Fig. 1G, H), which was much lower than that of cisplatin alone (Fig. 1C, IC_50_ = 10.14 µg/ml).

### Cisplatin and Doxycycline inhibit the invasion ability of epithelial ovarian cancer cells

The effect of cisplatin and doxycycline on the invasion ability of tumor cells was examined by an invasion assay. Firstly, we selected 1.5 µg/ml and 5 µg/ml cisplatin to treat SKOV3 and SKOV3/DDP cells respectively. Fig. S2A, B represented tumor cell invasion ability in the presence (c) or absence (d) of cisplatin in both SKOV3 and SKOV3/DDP cells. We found that cisplatin had an inhibitory effect on ovarian cells invasion ability. Then, we selected 10 µg/ml doxycycline to treat SKOV3 cells and 5 µg/ml doxycycline to treat SKOV3/DDP cells. Figure 2A, B represented tumor cell invasion ability in the presence (c) or absence (d) of doxycycline in both SKOV3 (Fig. 2A) and SKOV3/DDP (Fig. 2B) cells. For the first time we found that doxycycline could inhibit the invasion ability of both SKOV3 and SKOV3/DDP cells.

RETRACTED

**Figure 2:** Inhibition of doxycycline on epithelial ovarian cancer cells invasion. Cells were cultured in transwell with indicated doxycycline for 36/DDP cells by 4 and 2 folds respectively. a: 100 µl serum-free cell suspension (after cells attached) with doxycycline-treated (10 µg/ml) in coated insert filters; 500 µl serum-free RPMI-1640 medium with doxycycline (10 µg/ml) in the lower chambers, pictures were photographed from the upper side of the membranes. b: 100 µl serum-free cell suspension in coated insert filters; 500 µl serum-free RPMI-1640 medium in the lower chambers, pictures were photographed from the upper side of the membranes. c: 100 µl serum-free cell suspension (after cells attached) with doxycycline-treated (10 µg/ml) in coated insert filters; 500 µl 10%FBS/RPMI-1640 medium in the lower chambers, pictures were photographed from the lower side of the membranes. **d**: 100 µl serum-free cell suspension in coated insert filters; 500 µl 10%FBS/RPMI-1640 medium in the lower chambers, pictures were photographed from the lower side of the membranes. c/a represents the ratio of cells coming though the membrane of filter insert with doxycycline treatment. d/b represents the ratio of cells coming though the membrane of filter insert without doxycycline. C, D showed that Doxycycline inhibits sdf-1α-induced invasion in both cell lines and a moderate apoptosis induced by doxycycline in SKOV3/DDP cells and inhibition by doxycycline on SDF-1α secretion in SKOV3 cells. C: SDF-1α increased the invasion of SKOV3 cells by 9 folds which was inhibited by doxycycline (10 µg/ml). D: SDF-1α only increased the invasion of SKOV3/DDP cells by 1.5 folds which was inhibited by doxycycline (5 µg/ml). n = 3,*, *p*<0.05,**, *p*<0.01.

### Doxycycline inhibits SDF-1α-induced tumor cell invasion in ovarian cancer cells

SDF-1α is a member of chemokines and plays an important role in the metastasis of ovarian cancer [12]. In order to investigate whether SDF-1α could promote the invasive ability of ovarian cancer cells, we then changed the induced-factor (10% FBS) to SDF-1α (50 ng/ml). As shown in Fig. 2C, SDF-1α increased the invasion of SKOV3 cells by 9 folds, which could be significantly inhibited by doxycycline. While in SKOV3/DDP cells, SDF-1α in the same dose only increased the invasion ability by 1.5 times, which could also be inhibited by doxycycline (Fig. 2D).

### Doxycycline induces apoptosis of SKOV3/DDP but not of SKOV3 cells

The apoptotic ratio was tested in two cell lines after treatment with 5, 10 and 20 µg/ml doxycycline for 12 h. As shown in Figure 3A, doxycycline (20 µg/ml) increased apoptosis of SKOV3/DDP cells by 13 folds while had no effect on SKOV_3_ cells.

RETRACTED

**Figure 3:** A moderate apoptosis induced by doxycycline in SKOV3/DDP cells and inhibition by doxycycline on SDF-1α/CXCR4 axis in SKOV3 cells. A: Flow cytometric analysis showing the cell apoptosis after treatment with different concentrations of doxycycline for 6 h. 20 µg/ml doxycycline increased the apoptosis of SKOV3/DDP cells by 13 folds. B: ELISA analysis showing doxycycline (10 µg/ml) inhibited secretion of SDF-1α in SKOV3 cells in a time-dependent manner. Real-time PCR and Western blot analysis showing the effects of doxycycline on CXCR4 expression in both mRNA and protein levels in SKOV3 cells (C, E) and SKOV3/DDP cells (D, F). After treatment with doxycycline of indicated concentrations for 48 h, CXCR4 expression in both mRNA and protein levels were inhibited significantly in two cell lines. n = 3. *, *p*<0.05,**, *p*<0.01.

### Doxycycline inhibits SDF-1α secretion in SKOV3 cells, but not in SKOV3/DDP cells

As SDF-1α and its receptor CXCR4 play an important role in the process of tumor invasion and metastasis [13], we then carried out ELISA assay to determine whether doxycycline could inhibit the secretion of SDF-1α in two cell lines. The results showed that in SKOV3, SDF-1α secretion was significantly decreased by treatment of doxycycline in a time-dependent manner, with the minimal level observed at 180 min (Fig. 3B). However, secretion of SDF-1α was not detected in SKOV3/DDP.

### Doxycycline decreases CXCR4 mRNA and protein levels in SKOV3 and SKOV3/DDP cells

CXCR4 could be activated by SDF-1α and is the only one of 14 chemokine receptors expressed in a subset of tumor cells in ovarian neoplasms and primary ovarian tumors [14]. In our experiments, cells were treated with different concentrations of doxycycline for 48 h, then CXCR4 mRNA and protein levels were examined by Real-time PCR and western blot analysis. We found that doxycycline inhibited CXCR4 expression at both mRNA (Fig. 3C. D) and protein levels (Fig. 3E, F) in both SKOV3 and SKOV3/DDP cell lines.

### Cisplatin and Doxycycline inhibit cell viability through Akt and ERK pathways in SKOV3 but not in SKOV3/DDP cells

It has been reported that cisplatin resistance of human ovarian cancer is related to activation of PI3K/Akt and ERK1/2 signaling pathways [15]–[16], we then determined the potential involvement of these two pathways in cisplatin and doxycycline effects on ovarian cancer cell proliferation. After depleting Akt and ERK by siRNA (Fig. 4A, B), the MTT results showed that reduction of Akt and ERK expression could attenuate the inhibitory effect on proliferation when treated with cisplatin and doxycycline for 48 h in SKOV3 (Fig. 4C, D, G, H), but had no effect on proliferation of SKOV3/DDP cells (Fig. 4E, F, I, J).

RETRACTED

**Figure 4:** Cisplatin and Doxycycline inhibit cell viability through Akt and ERK pathways in SKOV3 but not in SKOV3/DDP cells. Reduction of Akt and ERK expression by Akt and ERK siRNA could attenuate the inhibitory effect on proliferation when treated with cisplatin and doxycycline for 48(C, D, G, H) but had no effect on proliferation in SKOV3/DDP cells (E, F, I, J) *, *p*<0.05; **, *p*<0.01.

### Doxycycline inhibits SDF-1α-induced activation of Akt or ERK in SKOV3 but not in SKOV3/DDP

In order to understand whether SDF-1α-induced Akt and/or ERK phosphorylation in two cell lines can be inhibited by doxycycline, we performed a series of experiments with pre-treatment. Firstly, we investigated the phosphorylation of Akt and ERK in SKOV3 after SDF-1α treatment (50 ng/ml) for different time (0, 2, 5, 10, 20, 40 min). As shown in Fig. 5A, B, SDF-1α stimulated Akt and ERK phosphorylation in a time-dependent manner. The Akt and ERK were significantly phosphorylated and reached a maximum at 10 or 20 min after SDF-1α treatment. The similar experiments were then carried out in SKOV3/DDP. Notably, there was no activation of Akt and ERK after treatment of SDF-1α (data not shown). Further, we shortened the treatment time to less than 10 min. We still did not find any activation of Akt (Fig. 5C) while ERK activation was increased from 0.5 min and reached a maximum at 1 min (Fig. 5D). Next, SKOV3 cells were pre-treated with doxycycline (0, 5, 10 µg/ml) for 3 h, and then were applied with SDF-1α (50 ng/ml) for 10 min. Inhibition of phosphor-Akt and phosphor-ERK levels was observed after application of 10 µg/ml doxycycline (Fig. 5E, F). Application of doxycycline alone had no effect. Similarly, SKOV3/DDP cells were pre-treated with the same dose of doxycycline for 3 h, and then treated with SDF-1α (50 ng/ml) for 1 min. Doxycycline had no effect on Akt activation (Fig. 5G). SDF-1α-induced ERK phosphorylation could not be blocked by doxycycline at the dose of 5 or 10 µg/ml. (Fig. 5H).

**Figure 5:** Western blot analysis showing the effects of doxycycline on SDF-1α-induced AKT/ERK phosphorylation in SKOV3 and SKOV3/DDP cell lines. After treatment of SDF-1α (50 ng/ml) for 0, 2, 5, 10, 20, 40 minutes, AKT (A) and ERK (B) phosphorylation in SKOV3 cells were augmented. When treated SKOV3/DDP with the same dose of SDF-1α for 0, 0.5, 1, 2, 5, 10 minutes, AKT phosphorylation (C) did not change, while ERK phosphorylation (D) was augmented significantly. Then, cells were pretreated with 0, 5, 10 µg/ml doxycycline for 3 h, then treated with SDF-1α (50 ng/ml) for 10 min (SKOV3) or 1 min (SKOV3/DDP), SDF-1α-induced AKT (E) and ERK (F) phosphorylation in SKOV3 cells were only inhibited when co-application with doxycycline at dose 10 µg/ml. In SKOV3/DDP cells, SDF-1α did not induce AKT phosphorylation (G) and enhanced ERK phosphorylation (H) could not be blocked by doxycycline at dose 5 or 10 µg/ml. n = 3. *, *p*<0.05, **, *p*<0.01, SDF-1α-treated groups *vs* control group. #, *p*<0.01, SDF-1α plus doxycycline co-treated groups *vs* SDF-1 treated groups.

RETRACTED

### Doxycycline upregulates pro-caspase-3 expression in SKOV3/DDP but not in SKOV3

Caspase-3 is an important mediator of apoptosis and could also be associated with chemoresistance of human ovarian cancer [17]. We then observed the changes in its expression in two cell lines after doxycycline treatment. Firstly, we compared Akt, ERK phosphorylation, CXCR4 and pro-caspase-3 expression between two cell lines. The results showed that there was no significant difference of Akt phosphorylation (Fig. 6A). ERK phosphorylation, CXCR4 and pro-caspase-3 expression in SKOV3/DDP were all lower than those in SKOV3 cells, respectively (Fig. 6B, C, D). Then, we treated two cell lines with 10 µg/ml doxycycline for different time (0, 0.5, 1, 2, 6, 12 h). As shown in Fig. 6E, pro-caspase-3 expression was increased significantly in SKOV3/DDP, while did not change in SKOV3.

**Figure 6:** Western blot analysis showing the upregulation of pro-caspase-3 expression by doxycycline in SKOV3/DDP cells but not in SKOV3 cells. Comparison of Akt, ERK, CXCR4 and pro-caspase-3 expression in two cell lines. There was no significant difference of Akt (A) phosphorylation in the two cell lines. ERK phosphorylation (B), CXCR4 (C) and pro-caspase-3 (D) expression in SKOV3/DDP cells were all lower than those in SKOV3 cells, respectively. Pro-caspase-3 expression was increased significantly by doxycycline treatment in SKOV3/DDP cells, while did not change in SKOV3 cells (E). n = 3. *, *p*<0.05, **, *p*<0.01.

### Doxycycline inhibits tumor xenograft

As an attempt to determine whether doxycycline contributes to tumor inhibition in vivo, we used SKOV3.ip xenograft model in nude mice (BALB/c-nu). Fourteen days after injection of tumor cells, doxycycline (i.p. injection) was then administrated (3 mg/d/per mice) for the next 7 days. Tumor diameters, mice body weights and ascites levels in tumor group and doxycycline-treated group were analyzed. Compared with those in tumor group, the tumor diameter and the volume of ascites were decreased significantly in doxycycline-treated group (Fig. 7B, C, F, G). The degree of aggregation of tumor cells in doxycycline-treated group (Fig. 7E) was less than that in tumor group (Fig. 7D). Moreover, the body weight in doxycycline-treated group was approach to that in control group (Fig. 7H).

RETRACTED

**Figure 7:** Inhibition of doxycycline on tumor diameter and malignant ascites in SKOV3.ip tumor xenograft. (A) From the outside appearance, the abdomen of tumor group was bulging obviously (b) than the one in control group (a) and the one in doxycycline-treated group (c). Doxycycline inhibited the growth of tumor xenograft (B, F) and the volume of malignant ascites (C, G) significantly in doxycycline-treated tumor mice compared with those of tumor mice. (D) HE staining showed that the degree of aggregation of tumor cells in doxycycline-treated group (E) was much less than that in tumor group. (H) The body weight in tumor group was significantly lower than those of either control group or doxycycline-treated group. n = 6. **, *p*<0.01.

## Discussion

Cisplatin is a chemotherapeutic drug for ovarian cancer. Besides the serious side effects, the cisplatin-resistance is also a big obstacle. Combination of some innocuous components with chemotherapy drugs is an emerging new strategy for cancer chemotherapy to further improve the efficacy and to minimize the side effects. Doxycycline is widely accepted as an antibiotic. In our experiments, we demonstrated that doxycycline not only has an inhibitory effect on ovarian cancer, but also can dramatically enhance the chemosensitivity to cisplatin.

However, the underlying mechanism is still unclear. Some researches have reported that the antitumor effect of doxycycline is associated with different levels of p53 in hepatocellular carcinoma [18]. Another study demonstrates that doxycycline can induce apoptosis in human pancreatic and colon cancer cells through caspase-dependent way [19]–[20]. Our findings, for the first time, showed that doxycycline inhibited the secretion of SDF-1α in SKOV3, while similar phenomenon was not observed in SKOV3/DDP cells. Further research showed that doxycycline inhibited expression of CXCR4 at both mRNA and protein levels, suggesting its effect might be at transcription level. Western-blot analysis also indicated that CXCR4 expression in SKOV3/DDP was 20% lower than that in SKOV3. These results suggested that SDF-1α/CXCR4 axis may have different roles in doxycycline effects in the two cell lines. Several explanations may contribute to this phenomenon: 1) Upon activation, CXCR4 can mediate tumor metastasis. Tumor cells entering the blood or lymphatic systems will migrate and adhere to areas with high expression of SDF-1α. Breast cancer cells follow this pattern of metastasis [21]. Here we describe that SKOV3 cells can secret SDF-1α and it has higher expression of CXCR4. Furthermore, SDF-1α promotes the invasion of SKOV3 by nine-fold. Based on these data, we postulated SDF-1/CXCR4 axis played a critical role in the metastasis of SKOV3 cells by increasing the adhesion capability of cancer cells, but SKOV3/DDP might not. 2) Some other studies indicated that epigenetic mechanisms involved in the negative regulation of SDF-1α or CXCR4 expression may be necessary for tumor metastasis. Typical modification of SDF-1α or CXCR4 such as DNA methylation is associated with the inactivation of tumor suppressors. There is evidence that methylation of the SDF-1α promoter in the colonic epithelium promotes metastasis of tumors in the colon [22]. Additionally, in pancreatic cancer, the CXCR4 promoter has been found to be regulated by DNA methylation, resulting in lower CXCR4 mRNA and protein levels [23]. Moreover, the C-terminal domain of CXCR4 also plays a major role in receptor regulation, particularly during the process of epithelial-to-mesenchymal transition (EMT). It has been reported that in MCF-7 mammary carcinoma cells, expression of the C-tail truncated mutant of CXCR4 results in a higher growth rate and EMT [24]. More importantly, recent evidence has indicated that processes of EMT plays a role in the development of chemoresistance [25]. We thus propose that the modulation, such as the methylation of SDF-1α or CXCR4 promoter, or the existence of C-tail truncated mutant of CXCR4, might happen in SKOV3/DDP cells, which lead to almost no detection of SDF-1α and lower expression of CXCR4 and the consequent chemoresistance. Further experiments are required to elucidate the underlying mechanisms.

RETRACTED

SDF-1α is also found in ascites fluid from ovarian cancer patients and promotes cancer development when binding to CXCR4 [26]. Accumulating data have implicated that SDF-1α/CXCR4 axis can cause mobilization of calcium, decrease of cyclic AMP with the cells and activation of multiple signaling pathways including PI3K/Akt and ERK1/2 [27]–[28], which are known to play important roles in the regulation of cell proliferation and survival. In our experiments, Akt and ERK1/2 pathways were involved in doxycycline effect on cell proliferation of SKOV3 but not of SKOV3/DDP cells. However, there was no induction of AKT phosphorylation in SKOV3/DDP by SDF-1α treatment. Furthermore, phosphorylation of ERK was enhanced in the earliest time points of 2 minutes and doxycycline (5 and 10 µg/ml) treatment had no inhibitory effect on it. These results indicate that SDF-1α/CXCR4-regulated Akt and ERK activations are involved in the regulation of SKOV3 cells by doxycycline but not in the SKOV3/DDP cells.

Previous studies have shown that caspase-3 activity is markedly reduced and apoptotic ratios are significantly lower in cisplatin-resistant (A2780/DDP, COC1/DDP) ovarian cancer cell lines [17]. In our study, the basic expression of caspase-3 was much lower in SKOV3/DDP than that in SKOV3. Doxycycline significantly increased the expression of pro-caspase-3 in SKOV3/DDP, but it had no effect on that in SKOV3. Combined with the MTT assay results showing that SKOV3/DDP cells were more sensitive to doxycycline, these results suggest that caspase-3 might be responsible for doxycycline sensitivity in SKOV3/DDP. The result, to some extent, was consistent with apoptosis assay that doxycycline caused moderate apoptosis in SKOV3/DDP, but had no significant effect on SKOV3. Therefore, caspase-3 might be new target for cisplatin resistance of SKOV3/DDP and making cells more sensitive to doxycycline, but the specific mechanism needs further study.

RETRACTED

In vivo experiments, the dose of 0.15 mg/g/day (a mice weight about 20 g in our experiment) for i.p. in mouse was equal to that of about 180 mg/day for an adult with oral administration. It has been reported doxycycline at a dose of 200 mg/day/person exhibits few side-effects [29].

In conclusion, our results experimentally showed that doxycycline can inhibit the progress of ovarian cancer and increase antitumor response of tumor cells to growth inhibition by cisplatin. From a mechanistic standpoint, doxycycline downregulates PI3K/Akt and ERK1/2 pathway through SDF-1α/CXCR4 axis in SKOV3 cells. In SKOV3/DDP, doxycycline upregulates the expression of pro-caspase-3, leading to the sensitization of cancer cells to doxycycline-induced inhibition of proliferation and increased apoptosis. The results provide a firm molecular basis for the pharmacologic effect underlying the use of doxycycline as a valuable therapeutic adjuvant. Given the safety of doxycycline, the present work should expedite the use of doxycycline in clinical trials.

## Supporting Information

Figure S1 **MTT tests showing the viability of ovarian cancer cells HO8910 incubated with indicated concentrations of cisplatin (A) and doxycycline (B) for 48 h.** Cell viability was inhibited in a dose-dependent manner by treatment with cisplatin and doxycycline. Then, HO8910 cells were treated with different concentrations of two drugs in the indicated drug administration sequences. C, D showed that co-treatment with cisplatin (1.0 µg/ml and 1.5 µg/ml) and doxycycline (7.5 or 10 µg/ml) had a significant grow inhibition in HO8910 cells compared with that of cisplatin treated alone. n = 9. *, *p*<0.05; **, *p*<0.01.
(TIF)

Figure S2 **Inhibition of cisplatin on epithelial ovarian cancer cells invasion.** Cells were cultured in transwell with indicated doxycycline for 36 h. Cells coming though the membrane of the filter insert and staying in the lower side represents an ability of invasion. A, B showed that doxycycline decreased the invasion of SKOV3 and SKOV3/DDP cells by 1.4 and 1.7 folds respectively. n = 3,*, *p*<0.05,**, *p*<0.01.
(TIF)

RETRACTED

## References

[1] JemalA, SiegelR, XuJ, WardE (2010) Cancer statistics. CA Cancer J Clin 60: 277–300.2061054310.3322/caac.20073

[2] BrayF, RenJS, MasuyerE, FerlayJ (2013) Global estimates of cancerprevalence for 27 sites in the adult population in 2008. Int J Cancer 132: 1133–1145.2275288110.1002/ijc.27711

[3] SuhDH, KimK, KimJW (2012) Major clinical research advances in gyneco-logic cancer in 2011. J Gynecol Oncol 23: 53–64.2235546810.3802/jgo.2012.23.1.53PMC3280068

[4] GubbelsJA, ClaussenN, KapurAK, ConnorJP, PatankarMS (2010) The detection, treatment, and biology of epithelial ovarian cancer. J Ovarian Res 3: 8.2035031310.1186/1757-2215-3-8PMC2856581

[5] BottoneMG, SoldaniC, VeneroniP, AvellaD, PisuM, et al (2008) Cell proliferation, apoptosis and mitochondrial damage in rat B50 neuronal cells after cisplatin treatment. Cell Proliferation 41 (3) 506–520.1839733710.1111/j.1365-2184.2008.00530.xPMC6496376

[6] MarshS (2009) Pharmacogenomics of Taxane/Platinum therapy in ovarian cancer. Int J Gynecol Cancer 2: 30–34.10.1111/IGC.0b013e3181c1051319955911

[7] JelovacD, ArmstrongDK (2011) Recent progress in the diagnosis and treatment of ovarian cancer. CA Cancer J Clin 61: 183–203.2152183010.3322/caac.20113PMC3576854

[8] ShenLC, ChenYK, LinLM, ShawSY (2010) Anti-invasion and anti-tumor growth effect of doxycycline treatment for human oral squamous-cell carcinoma–in vitro and in vivo studies. Oral Oncol 46 (3) 178–184.2003660410.1016/j.oraloncology.2009.11.013

[9] SunT, ZhaoN, NiCS, ZhaoXL, ZhangWZ, et al (2009) Doxycycline inhibits the adhesion and migration of melanoma cells by inhibiting the expression and phosphorylation of focal adhesion kinase (FAK). Cancer Lett 28; 285 (2) 141–150.10.1016/j.canlet.2009.05.00419482420

[10] TangH, SampathP, YanX, ThorneSH (2013) Potential for enhanced therapeutic activity of biological cancer therapies with doxycycline combination. Gene Ther doi:10.1038/gt. 2012.96 10.1038/gt.2012.96PMC362068123282955

[11] Han-junL, Li-yaW, Hai-naQ, Li-huaY, BurnstockG, et al (2011) P2Y2 receptor-mediated modulation of estrogen-induced proliferation of breast cancer cells. Molecular and Cellular Endocrinology 338: 28–37.2135627110.1016/j.mce.2011.02.014

[12] BarbieriE, BajettoA, FlorioT (2010) Role of chemokine network in the development and progression of ovarian cancer: a potential novel pharmacological target. J Oncol 426956.10.1155/2010/426956PMC279866920049170

RETRACTED

[13] BalkwillF (2004) Cancer and the chemokine network. Net Rev Cancer 4: 540–550.10.1038/nrc138815229479

[14] ScottonCJ, WilsonJL, MillikenD, StampG, BalkwillFR (2001) Epithelial cancer cell migration: a role for chemokine receptor? Cancer Res 61: 4961–4965.11431324

[15] NonakaM, ItamochiH, KawaguchiW, KudohA, SatoS, et al (2012) Activation of the mitogen-activated protein kinase kinase/extracellular signal-regulated kinase pathway overcomes cisplatin resistance in ovarian carcinoma cells. Int J Gynecol Cancer 22 (6) 922–929.2267298510.1097/IGC.0b013e31824f0b13

[16] YoonH, MinJK, LeeJW, KimDG, HongHJ (2011) Acquisition of chemoresistance in intrahepatic cholangiocarcinoma cells by activation of AKT and extracellular signal-regulated kinase (ERK)1/2. Biochem Biophys Res Commun 405 (3) 333–337.2113073110.1016/j.bbrc.2010.11.130

[17] YangX, ZhengF, XingH, GaoQ, WeiW, et al (2004) Resistance to chemotherapy-induced apoptosis via decreased caspase-3 activity and overexpression of antiapoptotic proteins in ovarian cancer. J Cancer Res Clin Oncol 130: 423–428.1515639810.1007/s00432-004-0556-9PMC12161855

[18] LaiPB, ChiTY, ChenGG (2007) Different levels of p53 induced either apoptosis or cell cycle arrest in a doxycycline-regulated hepatocellular carcinoma cell line in vitro. Apoptosis 12: 387–393.1719112610.1007/s10495-006-0571-1

[19] MouratidisPX, ColstonKW, DalgleishAG (2007) Doxycycline induces caspase-dependent apoptosis in human pancreatic cancer cells. Int J Cancer 120: 743–752.1713130810.1002/ijc.22303

[20] OnodaT, OnoT, DharDK, YamanoiA, NagasueN (2006) Tetracycline analogues (doxycyclinee and COL-3) induce caspase-dependent and -independent apoptosis in human colon cancer cells. Int J Cancer 118: 1309–1315.1615260410.1002/ijc.21447

[21] AllinenM, BeroukhimR, CaiL, BrennanC, Lahti-DomeniciJ, et al (2004) Molecular characterization of the tumor microenvironment in breast cancer. Cancer Cell 6: 17–32.1526113910.1016/j.ccr.2004.06.010

[22] WendtMK, JohanesenPA, Kang-DeckerN, BinionDG, ShahV, et al (2006) Silencing of epithelial CXCL12 expression by DNA hypermethylation promotes colonic carcinoma metastasis. Oncogene 25: 4986–4997.1656808810.1038/sj.onc.1209505PMC4610155

[23] SatoN, MatsubayashiH, Fukushima N GogginsM (2005) The chemokine receptor CXCR4 is regulated by DNA methylation in pancreatic cancer. Cancer Biol Ther 4: 70–76.1566213310.4161/cbt.4.1.1378

[24] UedaY, NeelNF, Schutyser E RamanD, RichmondA (2006) Deletion of the COOH-terminal domain of CXC chemokine receptor 4 leads to the down-regulation of cell-to-cell contact, enhanced motility and proliferation in breast carcinoma cells. Cancer Res 66: 5665–5675.1674070410.1158/0008-5472.CAN-05-3579PMC2664111

RETRACTED

[25] HayE (2005) The mesenchymal cell, its role in the embryo, and the remarkable signaling mechanisms that create it. Dev Dyn 233: 706–720.1593792910.1002/dvdy.20345

[26] MiyanishiN, SuzukiY, SimizuS, KuwabaraY, BannoK, et al (2010) Involvement of autocrine CXCL12/CXCR4 system in the regulation of ovarian carcinoma cell invasion. Biochem Biophys Res Commun 403: 154–159.2105934110.1016/j.bbrc.2010.11.007

[27] GanjuRK, BrubakerSA, Meyer J DuttP, YangY, et al (1998) The a-chemokine, stromal cell-derived factor-1a, binds to the transmembrane G-protein-coupled CXCR-4 receptor and activates multiple signal transduction pathways. J Biol Chem 273: 23169–23175.972254610.1074/jbc.273.36.23169

[28] SotsiosY, WhittakerGC, WestwickJ, WardSG (1999) The CXC chemokine stromal cell-derived factor activates a Gi-coupled phosphoinositide 3-kinase in T lymphocytes. J Immunol 163: 5954–5963.10570282

[29] SunBC, ZhangSW, QiLS, ZhangDF, GuoH, et al (2006) Study on the molecular mechanism of endostatin and doxycycline in suppressing melanoma growth. Zhonghua Bing Li Xue Za Zhi 35: 677–680.17374213

